# Developmental Genes and Regulatory Proteins, Domains of Cognitive Impairment in Schizophrenia Spectrum Psychosis and Implications for Antipsychotic Drug Discovery: The Example of Dysbindin-1 Isoforms and Beyond

**DOI:** 10.3389/fphar.2019.01638

**Published:** 2020-01-29

**Authors:** John L. Waddington, Xuechu Zhen, Colm M. P. O’Tuathaigh

**Affiliations:** ^1^ School of Pharmacy and Biomolecular Sciences, Royal College of Surgeons in Ireland, Dublin, Ireland; ^2^ Jiangsu Key Laboratory of Translational Research & Therapy for Neuro-Psychiatric Disorders and Department of Pharmacology, College of Pharmaceutical Sciences, Soochow University, Suzhou, China; ^3^ Medical Education Unit, School of Medicine, Brookfield Health Sciences Complex, University College Cork, Cork, Ireland

**Keywords:** cognitive deficits, developmental gene, schizophrenia, antipsychotic drug development, dysbindin-1

## Abstract

Alongside positive and negative symptomatology, deficits in working memory, attention, selective learning processes, and executive function have been widely documented in schizophrenia spectrum psychosis. These cognitive abnormalities are strongly associated with impairment across multiple function domains and are generally treatment-resistant. The DTNBP1 (dystrobrevin-binding protein-1) gene, encoding dysbindin, is considered a risk factor for schizophrenia and is associated with variation in cognitive function in both clinical and nonclinical samples. Downregulation of DTNBP1 expression in dorsolateral prefrontal cortex and hippocampal formation of patients with schizophrenia has been suggested to serve as a primary pathophysiological process. Described as a “hub,” dysbindin is an important regulatory protein that is linked with multiple complexes in the brain and is involved in a wide variety of functions implicated in neurodevelopment and neuroplasticity. The expression pattern of the various dysbindin isoforms (-1A, -1B, -1C) changes depending upon stage of brain development, tissue areas and subcellular localizations, and can involve interaction with different protein partners. We review evidence describing how sequence variation in DTNBP1 isoforms has been differentially associated with schizophrenia-associated symptoms. We discuss results linking these isoform proteins, and their interacting molecular partners, with cognitive dysfunction in schizophrenia, including evidence from drosophila through to genetic mouse models of dysbindin function. Finally, we discuss preclinical evidence investigating the antipsychotic potential of molecules that influence dysbindin expression and functionality. These studies, and other recent work that has extended this approach to other developmental regulators, may facilitate identification of novel molecular pathways leading to improved antipsychotic treatments.

## Introduction

### Schizophrenia, Cognitive Impairment, and Functional Disability

Schizophrenia is a complex psychiatric disorder that is the exemplar of a broader spectrum of psychotic illness in which interactive contributions from genetic and environmental factors play critical roles in etiology and pathobiology (Owen et al., 2016); hereafter, we use the term schizophrenia as shorthand for this spectrum of illness. In intimacy with positive, psychotic symptoms that define this spectrum, dysfunction in working memory, attention, processing speed, visual and verbal learning, reward-related learning, and prominent deficits in executive function have been extensively documented in schizophrenia (Kahn and Keefe, 2013). Impairment across these domains, in juxtaposition with negative symptoms, has long been accepted as core features of schizophrenia that contribute substantively to disability and are generally treatment refractory (Green et al., 2019).

Several authors have recommended inclusion of cognitive impairment in formal diagnostic criteria for this illness, as well as highlighting the need for research on developing new and more effective treatments to enhance cognitive abilities therein (Kahn and Keefe, 2013; Schaefer et al., 2013; Mark and Toulopoulou, 2016). Cognitive deficits associated with schizophrenia are observed in unaffected family members of individuals with the disorder (Toulopoulou et al., 2019) and the presence of schizophrenia-associated cognitive impairment in children can predict increased risk for the illness (Meier et al., 2014; Agnew-Blais et al., 2015).

### Schizophrenia, Cognitive Impairment, and Genetics

Twin studies continue to affirm a primary role for genetic factors in the etiology of schizophrenia (Hilker et al., 2018), in association and interaction with environmental adversities (Guloksuz et al., 2019). However, despite considerable endeavour during the past 20 years, genomic studies of schizophrenia have arguably failed to provide the expected answers, or have highlighted the difficulties in elucidating a complex, heterogeneous, and polygenic genetic architecture. The existing literature indicates contributions from multiple common and occasional rare variants that may interact in conferring risk for schizophrenia (Bergen et al., 2019; Weinberger, 2019). A key challenge in this field involves the translation of advances in our understanding of the genetics of schizophrenia and the mechanistic basis of these associations into tangible improvements in patient-centred care and antipsychotic drug discovery.

In support of a common disease-common allele hypothesis, whereby much of risk for schizophrenia is conferred *via* the cumulative effect of multiple common alleles, a landmark genome wide association study of more than 36,000 cases and over 113,000 controls identified 108 loci for common risk variants that achieved genome-wide significance (Schizophrenia Working Group of the Psychiatric Genomics Consortium, 2014). These risk variants are involved in several known processes, including synaptic plasticity and within the major histocompatibility complex, but also in as-yet unknown functions. In the most recent analysis completed by the same consortium, which involved 30,000 additional subjects, the number of GWAS-significant loci was expanded to 246 (Weinberger, 2019).

Polygenic risk scores (PRS) represent an aggregate measure of genetic risk as they consider the additive effects of all significant variation across multiple genes and regulatory areas across the entire genome (Jones et al., 2016; Xavier et al., 2018; Toulopoulou et al., 2019). The PRS is calculated by summing all the alleles (weighted by their individual odds ratios) that have been associated with an illness in the latest GWAS data set for that illness. In the most recent study of the effect of schizophrenia risk alleles on cognition (Richards et al., 2019), schizophrenia PRS were associated more strongly with case-control cognitive differences as opposed to variation within cases.

Copy number variants (CNVs), both rare *de novo* and inherited, make only a minor contribution to population risk variation despite larger effect sizes (Manolio et al., 2009; Malhotra and Sebat, 2012; Kotlar et al., 2015; Genovese et al., 2016). In schizophrenia, these rare variants are found at loci containing genes implicated in synaptic function as well as neurodevelopmental processes linked with glutamatergic function pathways (Kirov et al., 2012; Marshall et al., 2017). Genovese et al. (2016) reported that genes implicated in synaptic function potentially explained more than 70% of the exome enrichment in damaging ultra-rare variants that contribute to schizophrenia. Some authors have proposed a merging of common allele and rare variant mechanisms, suggesting that individuals with schizophrenia having well-characterized pathogenic CNVs also associate with an excess burden of common risk alleles (Tansey et al., 2016; Bergen et al., 2019).

More recent hypotheses suggest that the complex genetic architecture of schizophrenia may be better explained in terms of an “omnigenic” framework. This hypothesis (Boyle et al., 2017) posits that for complex traits such as schizophrenia, GWAS may identify genes more central to a disease process. However, these “core” genes function in a cellular network that is associated with the vastly more numerous other “peripheral” genes that have less evident relationship to disease but are able to influence the function of “core” genes. Indeed, recent evidence suggests in schizophrenia a “core” gene set that appears to contribute to risk to a greater extent than an omnigenic background effect (Rammos et al., 2019).

## Schizophrenia, Cognitive Impairment, and Variation in DTNBP1

Dysbindin-1 is a coiled-coil-containing protein encoded by DTNBP1 (Dystrobrevin Binding Protein 1, 6p22.3), a gene that has been linked with cognitive and anatomical endophenotypes in both patients with neuropsychiatric disorders as well as nonclinical samples (Ayalew et al., 2012; Wang et al., 2017; Savage et al., 2018). An initial report of genetic linkage to schizophrenia on chromosome 6p24-22 (Straub et al., 1995) was followed by multiple individual replications and confirmatory meta-analyses of DTNBP1 (Allen et al., 2008; Ayalew et al., 2012; Wang et al., 2017); any concern that such findings have not been prominent in GWAS studies to date (Farrell et al., 2015) must be juxtaposed with increasing recognition that GWAS cannot in itself be considered definitive on such issues (Tam et al., 2019; see also *Schizophrenia, Cognitive Impairment, and Genetics* above), and that the GWAS focus on diagnosis and symptom severity scores is likely to lead to neglect for genes specifically linked with cognitive dysfunction in schizophrenia. Additionally, the expression of dysbindin-1 and its isoforms is disrupted in brain tissue from schizophrenia patients (see *Schizophrenia Pathobiology and Dysbindin Isoforms* below). Importantly for issues to be considered further below, variations in DTNBP1 associated with schizophrenia (SNPs and haplotypes) are located in intron or promoter regions and almost all are located in the N-terminus of the gene (Guo et al., 2008).

Several studies have investigated the role of this gene in cognitive deficits of schizophrenia. For example, DTNBP1 haplotypes are associated with greater decline in IQ (Burdick et al., 2007) and impairment in spatial working memory (Donohoe et al., 2007; Donohoe et al., 2008; Donohoe et al., 2010) and attentional/vigilance (Baek et al., 2012), verbal and visual working memory and speed of processing (Varela-Gomez et al., 2015), as well as executive function (Scheggia et al., 2018). Such findings have been less evident on subdividing schizophrenia patients into cognitive-deficit and cognitive-sparing groups (Peters et al., 2008). Other studies have also failed to report a relationship between DTNBP1 variants and general tests of cognitive ability in patients with schizophrenia and first-degree relatives compared to controls (Strohmaier et al., 2010; Chow et al., 2018). Additionally, while some authors have shown that DTNBP1 variation in healthy controls and patients is associated with performance across a diverse range of cognitive tests (e.g. Burdick et al., 2006), a meta-analysis of 11 articles examining the relationship between dysbindin and general cognitive ability revealed only a modest relationship (Zhang et al., 2010). These results support involvement of the DTNBP1 gene in selective domains of cognition rather than non-specific cognitive ability (Luciano et al., 2009). Despite preliminary evidence to suggest dysbindin involvement in cognitive function in patients with brain tumours (Correa et al., 2016), there is a paucity of studies examining the role of dysbindin in other neurological and neuropsychiatric disorders where symptoms include cognitive dysfunction.

## Schizophrenia Pathobiology and Dysbindin Isoforms

Dysbindin expression levels vary across neuronal populations throughout the brain and are particularly abundant in the dentate gyrus of the hippocampal formation (Talbot et al., 2004; Talbot et al., 2006), with dysbindin localization in the CNS occurring in both neurons and, at comparable levels, in glia (Ghiani et al., 2009; Shao et al., 2011). DTNBP1 encodes for three major splice isoforms of dysbindin-1: 1A, 1B, and 1C. Dysbindin-1A is most highly concentrated in postsynaptic density fractions and dysbindin-1B is most abundant in synaptic vesicle fractions; similar to dysbindin-1A, dysbindin-1C is most highly concentrated in postsynaptic density fractions; nuclear localization has also been reported for dysbindin-1A and -1B (Oyama et al., 2009; Talbot et al., 2011).

Sequence variation might be a mechanism by which the function of DTNBP1 differs between schizophrenia cases and controls. In this scenario, instead of a simple incorrectly encoded protein, the amount of DTNBP1 expression may be affected. Indeed, it has been shown that variations in DTNBP1 affect its expression in the human brain (Bray et al., 2003; Bray et al., 2005; Bray et al., 2008).

The hippocampal formation plays a fundamental role in working and episodic memory, highlighting the possible role of dysbindin in cognitive processes that are believed to be critical to schizophrenia (Tamminga et al., 2010). Talbot et al. (2004) reported that schizophrenia patients show reduction of dysbindin-1 protein in the principal neurons of CA2 and CA3 and especially in the dentate gyrus of the hippocampal formation. A subsequent study from the same group reported that dysbindin proteins in the dentate gyrus are essentially present postsynaptically (Talbot et al., 2006). Talbot et al. (2011) then reported that in schizophrenia patients levels of dysbindin-1B and -1C, but not -1A, are decreased in the hippocampal formation, while levels of dysbindin-1A, but not -1B or -1C, are decreased in the superior temporal gyrus. Furthermore, transcripts encoding dysbindin-1B are upregulated in peripheral blood leukocytes of patients with schizophrenia relative to controls, with an intronic DTNBP1 variant associated with schizophrenia affecting splicing and leading to specific over-expression of dysbindin-1B (Xu et al., 2015).

Similarly to the hippocampal formation, the dorsolateral prefrontal cortex (DLPFC) is crucially involved in working and episodic memory, highlighting a further possible contribution of dysbindin to cognitive deficits encountered in schizophrenia (Lewis et al., 2008). Weickert et al. (2004) reported varying levels of DTNBP1 mRNA within the DLPFC, with higher expression found in layers IV and V; in DLPFC of schizophrenia patients decreases in DTNBP1 mRNA were reported in layers II, III, V and VI, but not in layers I and IV. Subsequently, decreases in DTNBP1 mRNA were reported in the hippocampal formation (Weickert et al., 2008). However, a subsequent study from the same team could not wholly confirm these findings (Fung et al., 2011). Tang et al. (2009) reported reductions in dysbindin-1C, but not in -1A or -1B, in DLPFC in the absence of changes in mRNA levels of the three isoforms. It should be noted that laminar-specific alterations in dysbindin mRNA and proteins may have escaped detection with the homogenate-based approach used in both studies (Tang et al., 2009; Fung et al., 2011). More recently, dysbindin-1B, but not -1A, protein levels were found to be higher in the DLPFC in schizophrenia (Konopaske et al., 2018).

## Schizophrenia, Neurodevelopment, Neuroplasticity, and Dysbindin

A wealth of epidemiological, clinical, and biological evidence now indicates that the origins of schizophrenia are to be found primarily in the early phases of fetal brain development: during this period a variety of factors, mainly genetic but also including environmental adversities, interact to disrupt brain morphogenesis (Waddington et al., 2012; Birnbaum and Weinberger, 2017); thereafter, endogenous and exogenous factors and processes can act to further “sculpt” brain development and maturation as a substrate from which the diagnostic symptoms and disabilities of clinical psychosis emerge, most typically during early adulthood (Waddington et al., 2012; Weinberger, 2017).

Regulation of brain development involves a multitude of genetic processes and associated proteins that act and interact sequentially to determine “normal” adult cerebral structure and function. Among these, dysbindin is one important regulator that is linked with multiple complexes in the brain and numerous diverse functions implicated in neurodevelopment and neuroplasticity. However, while the different dysbindin isoform proteins might interact with different partners, the majority of studies do not provide sufficient information to confirm or refute isoform-specific processes.

### Promotion of Cell Growth, Proliferation, and Antiapoptotic Effects

Dysbindin promotes activation of Akt (Numakawa et al., 2004), which mediates growth and proliferation of cells (Manning and Cantley, 2007). Akt has itself been proposed as a risk gene for schizophrenia and a target for antipsychotic drug development (Zheng et al., 2012; Enriquez-Barreto and Morales, 2016). Studies have reported that dysbindin is present in neurites and in axonal growth cones and that down regulation of dysbindin results in aberrant organisation of the actin cytoskeleton at the tips of neurites of differentiating cells, with shortening of such neurites (Kubota et al., 2009; Taneichi-Kuroda et al., 2009).

### BLOC-1 and Endosomal Trafficking

Dysbindin is a stable component of the multi-subunit complex BLOC-1 (biogenesis of lysosome-related organelles complex-1; Dell’Angelica, 2004; Li et al., 2004; Lee et al., 2012). Among the subunits of BLOC-1, dysbindin interacts directly with pallidin, MUTED, and snapin (Li et al., 2003; Starcevic and Dell’Angelica, 2004). Mice containing constitutive deletion of the pallidin gene show performance deficits in two different measures of recognition memory: the novel object recognition task and a measure of social novelty recognition (Spiegel et al., 2015).

Studies have also reported an association between markers at MUTED and schizophrenia (Straub et al., 2005; but see also Gerrish et al., 2009). Moreover, both dysbindin and MUTED siRNA increased cell surface dopamine (DA) D2 receptors (D2R) and blocked DA-induced D2R internalization in human and rat cells. In contrast, decreased dysbindin altered neither D1 receptors (D1R) levels nor their basal expression or DA-induced internalisation (Iizuka et al., 2007). Such an increase in D2R signalling could contribute to the imbalance in DAergic neurotransmission characteristic of schizophrenia, i.e., hyperfunction through D2R and attenuation of such hyperfunction by current D2R antagonist antipsychotics (McCutcheon et al., 2019).

A recent review has comprehensively addressed the relationship and interactions between BLOC-1 genes/proteins and cognitive phenotypes observed in neurodevelopmental disorders (Hartwig et al., 2018). The predominant theme is that BLOC-1 subunits in brain areas linked to cognitive functions are part of a more complex set of molecular interactions, including proteins implicated in schizophrenia such as disrupted-in-schizophrenia-1 and SNARE (Talbot, 2009; Hartwig et al., 2018).

### Dysbindin and Dystrophin-Associated Protein Complex

Dysbindin binds to the dystrobrevins, which are components of the dystrophin-associated protein complex (DPC) (Benson et al., 2001; but see also Nazarian et al., 2006). In the brain, several DPC-like complexes have been implicated in cognitive impairment commonly found in patients with Duchenne muscular dystrophy (DMD) (Blake and Kröger, 2000). Indeed, DPC is necessary for maturation and function of a subset of inhibitory synapses (Grady et al., 2006). Lack of dystrophin in the mdx mouse model of DMD produces an altered distribution of dysbindin in the brain, suggesting a role for dysbindin-1 in the cognitive impairment observed in DMD patients (Sillitoe et al., 2003).

## Nonisoform- and Isoform-Specific Genetic Mutation Models for Dysbindin-1 Function

### Drosophila Mutants

One dysbindin protein has been demonstrated in drosophila, known as CG6865-PA. While the amino acid sequence of its coiled-coil domain is closely related to that of all known orthologs of dysbindin, neither its N-terminal nor its C-terminal region is closely related to corresponding regions in any vertebrate dysbindin ortholog. CG6865-PA shares 28% amino acid identity with human dysbindin-1A (Guo et al., 2009). Drosophila dysbindin mutants demonstrate impaired neurotransmission, disrupted synaptic homeostasis, presynaptic and postsynaptic morphological alterations, and disruption in short term memory (Dickman and Davis, 2009; Cheli et al., 2010; Shao et al., 2011; Gokhale et al., 2015; Mullin et al., 2015; Gokhale et al., 2016).

Shao et al. (2011) reported that neuronal disruption of dysbindin function in drosophila was associated with hypoglutamatergic transmission and deficits in working memory, while disruption of dysbindin function in glial cells was associated with hyperdopaminergia and locomotor hyperactivity; this latter effects was mediated *via* a reduction in the protein Ebony, a glia-specific beta-alanyl biogenic amine synthetase involved in metabolic degradation of biogenic amines in the nervous system. This study reveals distinct functions of dysbindin in neurons and glial cells and highlights the potential of new therapeutics for schizophrenia that target glial cells (Bernstein et al., 2015). As reduction of dysbindin in drosophila impacts on short-term memory, dysbindin-dependent pathways may shed further light on the mechanisms of cognitive dysfunction in schizophrenia (Larimore et al., 2014).

### Mutant Mouse Models

Genetic mouse models enable etiologically related investigation of the pathophysiology of schizophrenia, providing means to advance target discovery to improve treatment for psychotic illness (O’Tuathaigh and Waddington, 2015). The development of new and effective drug therapies generally requires analysis of the intact brain in valid preclinical models, most commonly involving rodents (Dawson et al., 2015). Therefore, integrated research strategies for the delineation of animal models, based on characterization of cognitive deficits and underlying mechanisms, have considerable translational potential (Diamantopoulou and Gogos, 2019). In particular, based on the role of working memory in supporting a variety of cognitive abilities and its association with deficits in social and occupational functioning in schizophrenia, characterization of these processes in any mutant model is fundamental to understanding the relevance of the experimental model to cognitive dysfunction in this disorder.

While dysbindin-1A is highly conserved among vertebrates, there is no ortholog of human dysbindin-1B in mice; dysbindin-1C is a 270 amino acid protein in humans and a 271 amino acid protein in mice (Talbot, 2009). A spontaneous deletion mutation in DTNBP1 occurred in the DBA/2J strain, leading to complete absence of dysbindin-1A and 1C proteins in homozygous mice and reduced expression levels in heterozygous mice; the sandy (sdy) coat colour of homozygous mutants gives the strain its name (Swank et al., 1991). While the earliest studies were carried out in mice with the original DBA/2J background (sdy/DBA), the mutation has been transferred subsequently onto a C57BL/6J background (sdy/B6). DBA/2J mice are homozygous for at least six mutations, of which four are associated with neural impairments (Cox et al., 2009; Talbot, 2009). These appear to account for a number of auditory and visual deficits, when compared with C57BL/6 mice.

### Sandy Mice on a DBA/2J Background

Studies indicated abnormalities related to cognitive impairment (disturbance of long-delay recognition memory during an object recognition test) in homozygous sdy/DBA mice without abnormalities related to basal activity levels or anxiety (Feng et al., 2008). These authors also confirmed a previous finding of direct interaction with and decrease in the steady-state level of snapin (a SNAP-25 binding protein), suggesting an upstream regulatory role of dysbindin on neurotransmitter release *via* snapin. Takao et al. (2008) also reported cognitive deficits, including impairment in long-term memory retention (Barnes maze test) and in working memory (T-maze, forced alternation task). Bhardwaj et al. (2009) also demonstrated deficits in short-term memory (object recognition memory test) and stronger dependent memory for fearful events in sdy/DBA mice. In a subsequent study such mutants showed impaired recognition memory in the novel object recognition and social recognition paradigms (Spiegel et al., 2015).

Kobayashi et al. (2011) demonstrated hypersensitivity to both serotonergic and DAergic modulation of DG-to-CA3 signal transmission in 4-month-old to 6-month-old male homozygous sdy/DBA mice. These authors also reported decreased expression of D1R mRNA in the hippocampus that could contribute to changes in synaptic modulation. Jentsch et al. (2009) reported impaired glutamatergic transmission through potentially both presynaptic and postsynaptic mechanisms in the prefrontal cortex (PFC) of heterozygous and homozygous sdy/DBA mice. While dysbindin deletion appears to decrease glutamate release at the axon terminal, it may also result in an increase in excitability that might be due to reduction in neuronal dendritic branching and/or transmitter release in GABAergic interneurons. This study also reported homozygous sdy/DBA mice to show impairment in a spatial working memory task (delayed nonmatch-to-position test), with heterozygous mutants showing an intermediate level of performance. Collectively, these results suggest that dysbindin dysregulation might contribute to the cognitive symptoms of schizophrenia by decreasing glutamatergic transmission, at least in the prefrontal cortex.

### Sandy Mice on a C57BL/6J Background

Studies involving the sandy mouse on a C57BL6 background also show cognitive deficits. Cox et al. (2009) first reported impairment in spatial memory and/or initial learning and acquisition (Morris water maze) in sdy/B6 mice. Carlson et al. (2011) reported reductions in sdy/B6 mice of auditory-evoked response adaptation, prepulse inhibition, and evoked γ-activity, which is most frequently linked with disrupted inhibition and reduction in parvalbumin (PV)-positive interneuron activity. Indeed, subsequent analyses revealed reduction of fast-spiking GABAergic inhibition and fewer PV cells in the hippocampus of sdy/B6 mice.

As previously shown in sdy/DBA mice (Jentsch et al., 2009), homozygous sdy/B6 mice showed a decrease in working memory performance (delayed nonmatch-to-position test) compared to wildtypes; these results correlated with degree of expression of the NR1 subunit of the NMDA receptor. Other studies have shown an altered GluN2B-GluN2A switch in the hippocampus and cortex of dysbindin mutant mice (Sinclair et al., 2016). Genetic loss of dysbindin-1 expression has also been shown to impact on NMDA receptor-dependent synaptic plasticity in the hippocampus in both sdy/DBA and sdy/B6 mice (Glen et al., 2014). Another study demonstrated that loss of dysbindin-1 leads to reduced mGluR1 signalling in the hippocampus, which is associated with altered hippocampal synaptic plasticity in sdy/B6 mice (Bhardwaj et al., 2015). Overall, these results suggest a role for dysbindin in the regulation of NMDA and cognition that might be associated with cognitive deficits in schizophrenia.

Papaleo et al. (2012) reported differences in reference memory (T-maze) or a habituation/dishabituation task (olfactory discrimination test) in sdy/B6 mice, which demonstrated more rapid acquisition of a working memory task (T-maze) and overall worse performance on the same test under more demanding (proactive interference) or more stressful (transfer in a new cage) conditions relative to controls. Other data from the same group suggested that interval timing deficits may be a crucial component of abnormal cognition in sdy/B6 mice and that these deficits might be improved with increased training and experience (Carr et al., 2012).

Subsequent experiments were conducted to evaluate D2R modulation of these behavioral effects (Papaleo et al., 2012). While chronic D2R agonist administration did not affect acquisition in the working memory test, under more demanding conditions this treatment impaired working memory performance in a manner comparable to that observed in sdy/B6 mice. These authors also reported enhanced excitability and excitatory inputs to pyramidal neurons in medial-PFC (mPFC) layer II/III (the layers principally involved in intracortical projections), as well as decreased excitatory inputs to fast-spiking GABAergic neurons (Papaleo et al., 2012). DAergic modulation of excitatory synaptic transmission in layer II/III pyramidal neurons involves CaM-kinase-II (CaMKII)-dependent mechanisms that have been implicated in learning and memory processes (Gonzalez-Islas and Hablitz, 2003). While sdy/B6 mutants displayed lower CaMKII and CaMKKβ protein levels in mPFC, control mice chronically treated with a D2R agonist showed the same specific reductions (with no change in CaMKIV and CaMKKα levels; Papaleo et al., 2012). Overall, these results suggest that some effects of dysbindin on cognition, associated with changes in cortical activity and CaMK components of the mPFC, are induced *via* upregulation of D2R. Consistent with a dysbindin-associated increase in D2 receptors, dysbindin deficiency was associated with an antipsychotic-dependent increase in the ratio between the D2Short (D2S) and D2Long (D2L) isoforms in the PFC of mice, which is associated with potentiation of cortical presynaptic D2R signalling (Scheggia et al., 2018).

It has been proposed that DA signalling and PFC-dependent cognition follow an inverted U-shaped relationship, by which both inadequate or excessive DAergic signalling has a disruptive effect on cognitive performance that reflects an imbalance in dopamine D1/D2R activation (Vijayraghavan et al., 2007). Consistent with this hypothesis, Papaleo et al. (2014) investigated the effects on working memory performance of simultaneous disruption of dysbindin and the gene encoding the COMT enzyme, which plays a central role in the degradation of DA in PFC. They showed that while disruption of either dysbindin or COMT alone produced an improvement in working memory performance in the discrete paired-trial variable-delay T-maze task, mice with disruption of both genes demonstrated impaired working memory performance. These authors demonstrated a similar epistatic interaction on working memory performance and accompanying activation of PFC in humans. Based on the literature, the behavioral effects of this genetic interaction in both human and murine working memory paradigms reflect the effects of both genes on D1/D2R signalling in PFC. The same authors recently reported, in both mice and patients with schizophrenia, an interaction between functional variation in both dysbindin and D3R genes and working memory and executive function performance (Leggio et al., 2019). Specifically, simultaneous reduction of D3R and dysbindin function was associated with improved performance in tasks accessing these cognitive domains. It was shown that this epistatic interaction was associated with a shift in the balance between D2R and D3R receptor expression in the PFC, leading to an increase in D2R signalling in that brain region.

### Dysbindin-1A Mutant Mice

We have recently described the generation of a genetic mouse model with isoform-specific deletion of dysbindin-1A protein (Petit et al., 2017). Initial phenotypic characterization showed sexually dimorphic phenotypes, with female knockouts (KO) being more reactive to stressful situations and male KO showing increased exploration during initial exposure to a novel environment that may be related to some disruption in habituation and dysregulation of hippocampus-dependent working memory function. No effect of genotype was observed during acquisition or during performance in long-term (olfactory) memory or either a conventional spatial working memory task (spontaneous alternation) or a low-interference delay-dependent working memory task; however, in a high-interference task variant, male KO mutants showed impairment in vulnerability to interference (Petit et al., 2017).

### Dysbindin-1B Mutant Mice

Another recent study, which involved a transgenic mouse model expressing the human dysbindin-1B isoform, documented the presence of middle- and late-stage apoptosis in the hippocampus of dysbindin-1B mutants; in a T-maze alternation task, these mutants also showed deficits in working memory (Yang and Xu, 2017). Dysbindin-1B expression was also shown to impair spatial learning in the Morris water maze (Yang et al., 2016).

### Dysbindin Gain-of-Function Mutant Mice

A further study described the behavioral phenotype of a gain-of-function dysbindin mutant (Shintani et al., 2014). Specifically, these authors generated a transgenic model that expressed the human dysbindin-1A isoform. Such mutants displayed unaltered sensory or motor behavior and no changes in anxiety, sensorimotor gating, or exploratory behavior; they evidenced heightened locomotor responsivity to methamphetamine and upregulation and downregulation of several genes in PFC, including decreases in Arc and Egr2 expression.

### Spp Dysbindin Mutant Mice

Most recently, behavioral and cognitive phenotypes have been investigated in mice containing a single point mutation in the salt and pepper (spp) allele of DTNBP1 (Chang et al., 2018). While spp mutants did not exhibit any deficits in working memory (T-maze alternation task), some deficits in aspects of recognition memory performance were observed. These mice also demonstrated a reduction in the schizophrenia-associated SNAP-25 protein in PFC. No data are available regarding relative isoform expression in the brains of spp mutants.

### Dysbindin Mutation × Exposure to Environmental Risk Factors

Emphasis on genetic risk factors for schizophrenia should be tempered by evidence from investigations in twins (Hilker et al., 2018) and epidemiological studies indicating a role for environmental factors that may act both independently and *via* gene-environment interactions (Guloksuz et al., 2019). Therefore, animal models of neuropsychiatric disorders can and should investigate experimental induction of/exposure to nongenetic risk factors, including psychosocial stress and biological insults. Though there is some debate around common pathological mechanisms underlying the impact of such manipulations on schizophrenia-related phenotypes (Bradshaw and Korth, 2019), a combination of dysbindin gene mutation and postnatal exposure to Poly I:C (a model of immune activation in relation to schizophrenia) has been investigated. In sdy/B6 mice, exposure to Poly I:C resulted in deficits in prepulse inhibition and recognition memory, together with findings contrary to expectations, such as reduced locomotion; sdy/B6 mice treated with Poly I:C also displayed attenuated contextual and cue-dependent fear conditioning memory (Al-Shammari et al., 2018).

## Dysbindin-1 and Putative Treatment Strategies for Cognitive Dysfunction in Schizophrenia

Consistent with the proposed role for the D2R in the PFC in mediating the putative effects of dysbindin variation on higher order cognitive processes (Papaleo et al., 2012; Scheggia et al., 2018; Leggio et al., 2019), a series of elegant translational studies have shown that patients and mice with genetic variation associated with decreased dysbindin-1 expression demonstrate improved responsivity to the effects of antipsychotic medication on executive function (Scheggia et al., 2018). Mechanistic interrogation of this interaction revealed that the cognitive response to antipsychotics was mediated by enhanced presynaptic D2R in PFC (Scheggia et al., 2018). A subsequent study revealed a putative role for epistatic D3R-dysbindin-1 interaction and executive function deficits in schizophrenia, highlighting the viability of D3R modulation as a treatment target for cognitive dysfunction (Leggio et al., 2019).

As outlined above, dysbindin disruption has also been proposed to underlie cognitive impairment observed in patients with Duchenne muscular dystrophy. A recent study investigated the effects of treatment with the cacao flavonoid (-)-epicatechin on brain dysbindin levels in the mdx mutant, a genetic mouse model of Duchenne muscular dystrophy; such treatment partially reversed genotype-dependent reductions in protein levels of the dystrophin-associated protein complex as well as dysbindin protein in PFC (Estrada-Mena et al., 2017). It was not reported whether this partial recovery was also observed at a behavioral level.

Investigation of transcriptional responses of developing hippocampal neurons in sdy/B6 mutants revealed not only the characteristic GABAergic interneuron deficiency but also changes in expression of the cation-chloride cotransporters NKCC1 and KCC2 during hippocampal development (Larimore et al., 2017). NKCC1 and KCC2 expression changes have been documented in the brains of patients with schizophrenia (Hyde et al., 2011; Sullivan et al., 2015) and NKCC1 agents, including the NKCC1 chloride antagonist bumetanide, have been studied in schizophrenia. Bumetanide reduced hallucinations in a case of schizophrenia (Lemonnier et al., 2016) and in a randomized, double-blind placebo-controlled clinical trial bumetanide treatment reduced hallucinations (Rahmanzadeh et al., 2017a) but did not exert broad antipsychotic activity (Rahmanzadeh et al., 2017b); cognition was not specifically investigated.

Consistent with the observed involvement of dysbindin in hippocampal and PFC glutamatergic function, a recent study investigated the impact of pharmacological enhancement of endogenous levels of brain-derived neurotrophic factor (BDNF) on dysbindin-related reduction of presynaptic calcium levels in PFC and social recognition memory in sdy/B6 mice (Saggu et al., 2013). Systemic treatment with fingolimod, a sphingosine 1-phosphate receptor modulator that has been shown to increase endogenous BDNF levels, attenuated deficits in recognition memory and sociability and in presynaptic calcium and BDNF levels in the PFC of sdy/B6 mice (Becker-Krail et al., 2017). BDNF levels in schizophrenia patients have been associated with impairment across multiple cognitive domains (Man et al., 2018; Yang et al., 2019). A recent review has highlighted that the BDNF gene should be prioritised for pharmacogenetic research into antipsychotic drugs and potential relevance to treatment response and adverse effects (Han and Deng, 2018).

Similarly, administration of CDPPB, a positive allosteric modulator of MGluR5, restored short-term recognition and spatial memory deficits (Morris water maze) in sdy/B6 mice (Bhardwaj et al., 2015). Given their effects on glutamatergic signalling, and particularly on NMDA receptor activity, MGluR5 modulators have been suggested to represent promising treatment targets for neuropsychiatric disorders that are characterized by cognitive deficits.

Expression of SREBP1, a sterol regulatory element binding protein (SREBP) that regulates the expression of genes implicated in biosynthesis of fatty acids, cholesterol, triglycerides, and phospholipids, is reduced in sdy/B6 mice and in schizophrenia patients; activation of SREBP1 and Arc, a protein implicated in memory and cognition, is reduced in sdy/B6 mice and both of these deficits were restored by treatment with clozapine, suggesting a link with cognitive dysfunction (Chen et al., 2016).

## Dysbindin-1 and Beyond

Given the indicated role for dysbindin-1 in the pathophysiology of schizophrenia and associated cognitive impairment, it will be heuristic to search for drug targets and molecules that might influence its expression and functionality. Those studies that indicate relationships between dysbindin-1 function, neuronal and behavioral processes associated with the pathobiology of psychotic illness and responsivity to current D2R antagonist antipsychotic drugs are particularly provocative in this regard; this is because they offer the prospect of clues to identifying non-DAergic mechanisms of antipsychotic activity. Importantly, these concepts generalize beyond dysbindin-1 to other developmental regulators. For example, in addition to identifying a role for dysbindin-1A in the regulation of schizophrenia-related behavioral processes, including specialised delay/interference-dependent working memory (Petit et al., 2017), we have recently identified a role for the developmental gene and regulatory protein neuregulin-1 (NRG1) in a triad with miRNA-143 and D2R that was revealed through investigation of schizophrenia-related behavioral abnormalities induced by phencyclidine; miRNA-143 directly targeted to the 3’ un-translated region of NRG1 mRNA to reduce protein expression of NRG1 and the D2R modulated expression of NRG1 in PFC (Wang et al., 2019).

The issues reviewed above constitute a substantive basis for such a search. Furthermore, they offer tantalising glimpses into mechanisms and putative target sites relating to DTNBP1/dysbindin-1A and how these concepts might generalize to a broader spectrum of developmental genes and regulatory proteins implicated in the pathobiology of schizophrenia spectrum psychosis.

## Author Contributions

JW, XZ, and CO’T reviewed the relevant literature and wrote this paper. JW, XZ, and CO’T revised the manuscript. All the authors listed agreed to the publication of this paper.

## Funding

This work was supported by Science Foundation Ireland through grant 07/IN.1/B960.

## Conflict of Interest

The authors declare that the research was conducted in the absence of any commercial or financial relationships that could be construed as a potential conflict of interest.

## References

[B1] Agnew-BlaisJ. C.BukaS. L.FitzmauriceG. M.SmollerJ. W.GoldsteinJ. M.SeidmanL. J. (2015). Early childhood IQ trajectories in individuals later developing schizophrenia and affective psychoses in the New England family studies. Schizophr. Bull. 41, 817–823. 10.1093/schbul/sbv027 25904723PMC4466188

[B2] AllenN. C.BagadeS.McQueenM. B.IoannidisJ. P.KavvouraF. K.KhouryM. J. (2008). Systematic meta-analyses and field synopsis of genetic association studies in schizophrenia: the SzGene database. Nat. Genet. 40, 827–834. 10.1038/ng.171 18583979

[B3] Al-ShammariA. R.BhardwajS. K.MusaelyanK.SrivastavaL. K.SzeleF. G. (2018). Schizophrenia-related dysbindin-1 gene is required for innate immune response and homeostasis in the developing subventricular zone. NPJ Schizophr. 4, 15. 10.1038/s41537-018-0057-5 30038210PMC6056426

[B4] AyalewM.Le-NiculescuH.LeveyD. F.JainN.ChangalaB.PatelS. D. (2012). Convergent functional genomics of schizophrenia: from comprehensive understanding to genetic risk prediction. Mol. Psychiatry 17, 887–905. 10.1038/mp.2012.37 22584867PMC3427857

[B5] BaekJ. H.KimJ. S.RyuS.OhS.NohJ.LeeW. K. (2012). Association of genetic variations in DTNBP1 with cognitive function in schizophrenia patients and healthy subjects. Am. J. Med. Genet. Part B: Neuropsychiatr. Genet. 7, 841–849. 10.1002/ajmg.b.32091 22911901

[B6] Becker-KrailD.FarrandA. Q.BogerH. A.LavinA. (2017). Effects of fingolimod administration in a genetic model of cognitive deficits. J. Neurosci. Res. 95, 1174–1181. 10.1002/jnr.23799 27439747PMC6636312

[B7] BensonM. A.NeweyS. E.Martin-RendonE.HawkesR.BlakeD. J. (2001). Dysbindin, a novel coiled-coil-containing protein that interacts with the dystrobrevins in muscle and brain. J. Biol. Chem. 276, 24232–24241. 10.1074/jbc.M010418200 11316798

[B8] BergenS. E.PlonerA.HowriganD.O’DonovanM. C.SmollerJ. W. (2019). CNV Analysis Group and the Schizophrenia Working Group of the Psychiatric Genomics Consortium, Joint contributions of rare copy number variants and common SNPs to risk for schizophrenia. Am. J. Psychiatry 176, 29–35. 10.1176/appi.ajp.2018.17040467 30392412PMC6408268

[B9] BernsteinH. G.SteinerJ.GuestP. C.DobrowolnyH.BogertsB. (2015). Glial cells as key players in schizophrenia pathology: recent insights and concepts of therapy. Schizophr. Res. 161, 4–18. 10.1016/j.schres.2014.03.035 24948484

[B10] BhardwajS. K.BaharnooriM.Sharif-AskariB.KamathA.WilliamsS.SrivastavaL. K. (2009). Behavioral characterization of dysbindin-1 deficient sandy mice. Behav. Brain Res. 197, 435–441. 10.1016/j.bbr.2008.10.011 18984010

[B11] BhardwajS. K.RyanR. T.WongT. P.SrivastavaL. K. (2015). Loss of dysbindin-1, a risk gene for schizophrenia, leads to impaired group 1 metabotropic glutamate receptor function in mice. Front. Behav. Neurosci. 9, 72. 10.3389/fnbeh.2015.00072 25859193PMC4374471

[B12] BirnbaumR.WeinbergerD. R. (2017). Genetic insights into the neurodevelopmental origins of schizophrenia. Nat. Rev. Neurosci. 18, 727–740. 10.1038/nrn.2017.125 29070826

[B13] BlakeD. J.KrögerS. (2000). The neurobiology of Duchenne muscular dystrophy: learning lessons from muscle? Trends Neurosci. 23, 92–99. 10.1016/s0166-2236(99)01510-6 10675908

[B14] BoyleE. A.LiY. I.PritchardJ. K. (2017). An expanded view of complex traits: from polygenic to omnigenic. Cell 169, 1177–1186. 10.1016/j.cell.2017.05.038 28622505PMC5536862

[B15] BradshawN. J.KorthC. (2019). Protein misassembly and aggregation as potential convergence points for nongenetic causes of chronic mental illness. Mol. Psychiatry 24, 936–951. 10.1038/s41380-018-0133-2 30089789

[B16] BrayN. J.BucklandP. R.OwenM. J.O’DonovanM. C. (2003). Cis-acting variation in the expression of a high proportion of genes in human brain. Hum. Genet. 113, 149–153. 10.1007/s00439-003-0956-y 12728311

[B17] BrayN. J.PreeceA.WilliamsN. M.MoskvinaV.BucklandP. R.OwenM. J. (2005). Haplotypes at the dystrobrevin binding protein 1 (DTNBP1) gene locus mediate risk for schizophrenia through reduced DTNBP1 expression. Hum. Mol. Genet. 14, 1947–1954. 10.1093/hmg/ddi199 15917270

[B18] BrayN. J.HolmansP. A.van den BreeM. B.JonesL.EllistonL. A.HughesG. (2008). Cis-and trans-loci influence expression of the schizophrenia susceptibility gene DTNBP1. Hum. Mol. Genet. 17, 1169–1174. 10.1093/hmg/ddn006 18182443

[B19] BurdickK. E.LenczT.FunkeB.FinnC. T.SzeszkoP. R.KaneJ. M. (2006). Genetic variation in DTNBP1 influences general cognitive ability. Hum. Mol. Genet. 15, 1563–1568. 10.1093/hmg/ddi48 16415041

[B20] BurdickK. E.GoldbergT. E.FunkeB.BatesJ. A.LenczT.KucherlapatiR. (2007). DTNBP1 genotype influences cognitive decline in schizophrenia. Schizophr. Res. 89, 169–172. 10.1016/j.schres.2006.09.008 17074466PMC1828039

[B21] CarlsonG. C.TalbotK.HaleneT. B.GandalM. J.KaziH. A.SchlosserL. (2011). Dysbindin-1 mutant mice implicate reduced fast-phasic inhibition as a final common disease mechanism in schizophrenia. Proc. Natl. Acad. Sci. U.S.A. 108, E962–E970. 10.1073/pnas.1109625108 21969553PMC3203764

[B22] CarrG. V.JenkinsK. A.WeinbergerD. R.PapaleoF. (2012). Loss of dysbindin-1 in mice impairs reward-based operant learning by increasing impulsive and compulsive behavior. Behav. Brain Res. 241, 173–184. 10.1016/j.bbr.2012.12.021 23261874PMC3556458

[B23] ChangE. H.FernandoK.YeungL. W. E.BarbariK.ChandonT. S.MalhotraA. K. (2018). Single point mutation on the gene encoding dysbindin results in recognition deficits. Genes Brain Behav. 17, e12449. 10.1111/gbb.12449 29227583

[B24] CheliV. T.DanielsR. W.GodoyR.HoyleD. J.KandacharV.StarcevicM. (2010). Genetic modifiers of abnormal organelle biogenesis in a Drosophila model of BLOC-1 deficiency. Hum. Mol. Genet. 19, 861–878. 10.1093/hmg/ddp555 20015953PMC2816613

[B25] ChenY.BangS.McMullenM. F.KaziH.TalbotK.HoM. X. (2016). Neuronal activity-induced sterol regulatory element binding protein-1 (SREBP1) is disrupted in dysbindin-null mice-potential link to cognitive impairment in schizophrenia. Mol. Neurobiol. 54, 1699–1709. 10.1007/s12035-016-9773-x 26873854PMC4982840

[B26] ChowT. J.TeeS. F.LohS. Y.YongH. S.Abu BakarA. K.TangP. Y. (2018). Variants in ZNF804A and DTNBP1 assessed for cognitive impairment in schizophrenia using a multiplex family-based approach. Psychiatry Res. 270, 1166–1167. 10.1016/j.psychres.2018.04.051 29754893

[B27] CorreaD. D.SatagopanJ.CheungK.AroraA. K.Kryza-LacombeM.XuY. (2016). COMT, BDNF, and DTNBP1 polymorphisms and cognitive functions in patients with brain tumors. Neuro-Oncol. 18, 1425–1433. 10.1093/neuonc/now057 27091610PMC5035520

[B28] CoxM.TuckerA.TangJ.TalbotK.RicherD.YehL. (2009). Neurobehavioral abnormalities in the dysbindin-1 mutant, sandy, on a C57BL/6J genetic background. Genes Brain Behav. 8, 390–397. 10.1111/j.1601-183X.2009.00477.x 19220483PMC2774142

[B29] DawsonN.MorrisB. J.PrattJ. A. (2015). Functional brain connectivity phenotypes for schizophrenia drug discovery. J. Psychopharmacol. 29, 169–177. 10.1177/0269881114563635 25567554

[B30] Dell’AngelicaE. C. (2004). The building BLOC(k)s of lysosomes and related organelles. Curr. Op. Cell Biol. 16, 458–464. 10.1016/j.ceb.2004.05.001 15261680

[B31] DiamantopoulouA.GogosJ. A. (2019). Neurocognitive and perceptual processing in genetic mouse models of schizophrenia: emerging lessons. Neuroscientist Jan 17. 1073858418819435 10.1177/107385841881943530654694

[B32] DickmanD. K.DavisG. W. (2009). The schizophrenia susceptibility gene dysbindin controls synaptic homeostasis. Science 326, 1127–1130. 10.1126/science.1179685 19965435PMC3063306

[B33] DonohoeG.MorrisD. W.ClarkeS.McGheeK. A.SchwaigerS.NangleJ. M. (2007). Variance in neurocognitive performance is associated with dysbindin-1 in schizophrenia: a preliminary study. Neuropsychologia 45, 454–458. 10.1016/j.neuropsychologia.2006.06.016 16930638

[B34] DonohoeG.MorrisD. W.De SanctisP.MagnoE.MontesiJ. L.GaravanH. P. (2008). Early visual processing deficits in dysbindin-associated schizophrenia. Biol. Psychiatry 63, 484–489. 10.1016/j.biopsych.2007.07.022 17945199

[B35] DonohoeG.FrodlT.MorrisD.SpoletiniI.CannonD. M.CherubiniA. (2010). Reduced occipital and prefrontal brain volumes in dysbindin-associated schizophrenia. Neuropsychopharmacology 35, 368–373. 10.1038/npp.2009.140 19794403PMC3055383

[B36] Enriquez-BarretoL.MoralesM. (2016). The PI3K signaling pathway as a pharmacological target in Autism related disorders and Schizophrenia. Mol. Cell Ther. 4, 2. 10.1186/s40591-016-0047-9 26877878PMC4751644

[B37] Estrada-MenaF. J.RodriguezA.Mendoza-LorenzoP.Neri-GomezT.Manjarrez-GutierrezG.Perez-OrtizA. C. (2017). Effects of (-)-epicatechin on frontal cortex DAPC and dysbindin of the mdx mice. Neurosci. Lett. 658, 142–149. 10.1016/j.neulet.2017.08.056 28855126

[B38] FarrellM. S.WergeT.SklarP.OwenM. J.OphoffR. A.O’DonovanM. C. (2015). Evaluating historical candidate genes for schizophrenia. Mol. Psychiatry 20, 555–562. 10.1038/mp.2015.16 25754081PMC4414705

[B39] FengY.-Q.ZhouZ.-Y.HeX.WangH.GuoX.-L.HaoC.-J. (2008). Dysbindin deficiency in sandy mice causes reduction of snapin and displays behaviors related to schizophrenia. Schizophr. Res. 106, 218–228. 10.1016/j.schres.2008.07.018 18774265

[B40] FungS. J.SivagnanasundaramS.WeickertC. S. (2011). Lack of change in markers of presynatic terminal abundance alongside subtle reductions in markers of presynaptic terminal plasticity in prefrontal cortex of schizophrenia patients. Biol. Psychiatry 69, 71–79. 10.1016/j.biopsych.2010.09.036 21145444PMC3001685

[B41] GenoveseG.FromerM.StahlE. A.RuderferD. M.ChambertK.LandénM. (2016). Increased burden of ultra-rare protein-altering variants among 4,877 individuals with schizophrenia. Nat. Neurosci. 19, 1433–1441. 10.1038/nn.4402 27694994PMC5104192

[B42] GerrishA.WilliamsH.MoskvinaV.OwenM. J.O’DonovanM. C.WilliamsN. M. (2009). An examination of MUTED as a schizophrenia susceptibility gene. Schizophr. Res. 107, 110–111. 10.1016/j.schres.2008.08.011 18815010

[B43] GhianiC.StarcevicM.Rodriguez-FernandezI.NazarianR.CheliV.ChanL. (2009). The dysbindin-containing complex (BLOC-1) in brain: developmental regulation, interaction with SNARE proteins and role in neurite outgrowth. Mol. Psychiatry 15, 204–215. 10.1038/mp.2009.58 PMC281121319546860

[B44] GlenW.B.JrHorowitzB.CarlsonG. C.CannonT. D.TalbotK.JentschJ. D. (2014). Dysbindin-1 loss compromises NMDAR-dependent synaptic plasticity and contextual fear conditioning. Hippocampus 24, 204–213. 10.1002/hipo.22215 24446171PMC3937842

[B45] GokhaleA.MullinA. P.ZlaticS. A.EasleyC. A.4thMerrittM. E.RajN. (2015). The N-ethylmaleimide-sensitive factor and dysbindin interact to modulate synaptic plasticity. J. Neurosci. 35, 7643–7653. 10.1523/JNEUROSCI.4724-14.2015 25972187PMC4429160

[B46] GokhaleA.HartwigC.FreemanA. H.DasR.ZlaticS. A.VisteinR. (2016). The proteome of BLOC-1 genetic defects identifies the Arp2/3 Actin polymerization complex to function downstream of the schizophrenia susceptibility factor dysbindin at the synapse. J. Neurosci. 36, 12393–12411. 10.1523/JNEUROSCI.1321-16.2016 27927957PMC5148228

[B47] Gonzalez-IslasC.HablitzJ. J. (2003). Dopamine enhances EPSCs in layer II-III pyramidal neurons in rat prefrontal cortex. J. Neurosci. 23, 867–875. 10.1523/JNEUROSCI.23-03-00867.2003 12574415PMC6741914

[B48] GradyR. M.WozniakD. F.OhlemillerK. K.SanesJ. R. (2006). Cerebellar synaptic defects and abnormal motor behavior in mice lacking α-and β-dystrobrevin. J. Neurosci. 26, 2841–2851. 10.1523/JNEUROSCI.4823-05.2006 16540561PMC6673965

[B49] GreenM. F.HoranW. P.LeeJ. (2019). Nonsocial and social cognition in schizophrenia: current evidence and future directions. World Psychiatry 18, 146–161. 10.1002/wps.20624 31059632PMC6502429

[B50] GuloksuzS.PriesL. K.DelespaulP.KenisG.LuykxJ. J.LinB. D. (2019). Examining the independent and joint effects of molecular genetic liability and environmental exposures in schizophrenia: results from the EUGEI study. World Psychiatry 18, 173–182. 10.1002/wps.20629 31059627PMC6502485

[B51] GuoA.SunJ.RileyB.ThiseltonD.KendlerK.ZhaoZ. (2008). The dystrobrevin-binding protein 1 gene: features and networks. Mol. Psychiatry 14, 18–29. 10.1038/mp.2008.88 18663367PMC2859304

[B52] GuoA. Y.SunJ.RileyB. P.ThiseltonD. L.KendlerK. S.ZhaoZ. (2009). The dystrobrevin-binding protein 1 gene: features and networks. Mol. Psychiatry. 14, 18–29. 10.1038/mp.2008.88 18663367PMC2859304

[B53] HanM.DengC. (2018). BDNF as a pharmacogenetic target for antipsychotic treatment of schizophrenia. Neurosci. Lett. 9, 133870. 10.1016/j.neulet.2018.10.015 30312750

[B54] HartwigC.MonisW. J.ChenX.DickmanD. K.PazourG. J.FaundezV. (2018). Neurodevelopmental disease mechanisms, primary cilia, and endosomes converge on the BLOC-1 and BORC complexes. Dev. Neurobiol. 78, 311–330. 10.1002/dneu.22542 28986965PMC5816705

[B55] HilkerR.HeleniusD.FagerlundB.SkyttheA.ChristensenK.WergeT. M. (2018). Heritability of schizophrenia and schizophrenia spectrum based on the nationwide Danish twin register. Biol. Psychiatry 83, 492–498. 10.1016/j.biopsych.2017.08.017 28987712

[B56] HydeT. M.LipskaB. K.AliT.MathewS. V.LawA. J.MetitiriO. E. (2011). Expression of GABA signaling molecules KCC2, NKCC1, and GAD1 in cortical development and schizophrenia. J. Neurosci. 31, 11088–11095. 10.1523/JNEUROSCI.1234-11.2011 21795557PMC3758549

[B57] IizukaY.SeiY.WeinbergerD. R.StraubR. E. (2007). Evidence that the BLOC-1 protein dysbindin modulates dopamine D2 receptor internalization and signaling but not D1 internalization. J. Neurosci. 27, 12390–12395. 10.1523/JNEUROSCI.1689-07.2007 17989303PMC6673263

[B58] JentschJ. D.Trantham-DavidsonH.JairlC.TinsleyM.CannonT. D.LavinA. (2009). Dysbindin modulates prefrontal cortical glutamatergic circuits and working memory function in mice. Neuropsychopharmacology 34, 2601–2608. 10.1038/npp.2009.90 19641486PMC2762021

[B59] JonesH. J.StergiakouliE.TanseyK. E.HubbardL.HeronJ.CannonM. (2016). Phenotypic manifestation of genetic risk for schizophrenia during adolescence in the general population. JAMA Psychiatry 73, 221–228. 10.1001/jamapsychiatry.2015.3058 26818099PMC5024747

[B60] KahnR. S.KeefeR. S. (2013). Schizophrenia is a cognitive illness: time for a change in focus. JAMA Psychiatry 70, 1107–1112. 10.1001/jamapsychiatry.2013.155 23925787

[B61] KirovG.PocklingtonA. J.HolmansP.IvanovD.IkedaM.RuderferD. (2012). De novo CNV analysis implicates specific abnormalities of postsynaptic signalling complexes in the pathogenesis of schizophrenia. Mol. Psychiatry 17, 142–153. 10.1038/mp.2011.154 22083728PMC3603134

[B62] KobayashiK.Umeda-YanoS.YamamoriH.TakedaM.SuzukiH.HashimotoR. (2011). Correlated alterations in serotonergic and dopaminergic modulations at the hippocampal mossy fiber synapse in mice lacking dysbindin. PloS One 6, e18113. 10.1371/journal.pone.0018113 21448290PMC3063243

[B63] KonopaskeG. T.BaluD. T.PrestiK. T.ChanG.BenesF. M.CoyleJ. T. (2018). Dysbindin-1 contributes to prefrontal cortical dendritic arbor pathology in schizophrenia. Schizophr. Res. 201, 270–277. 10.1016/j.schres.2018.04.042 29759351PMC6230503

[B64] KotlarA. V.MercerK. B.ZwickM. E.MulleJ. G. (2015). New discoveries in schizophrenia genetics reveal neurobiological pathways: a review of recent findings. Eur. J. Med. Genet. 58, 704–714. 10.1016/j.ejmg.2015.10.008 26493318PMC4679408

[B65] KubotaK.KumamotoN.MatsuzakiS.HashimotoR.HattoriT.OkudaH. (2009). Dysbindin engages in c-Jun N-terminal kinase activity and cytoskeletal organization. Biochem. Biophys. Res. Commun. 379, 191–195. 10.1016/j.bbrc.2008.12.017 19094965

[B66] LarimoreJ.ZlaticS. A.GokhaleA.TornieriK.SingletonK. S.MullinA. P. (2014). Mutations in the BLOC-1 subunits dysbindin and muted generate divergent and dosage-dependent phenotypes. J. Biol. Chem. 289, 14291–14300. 10.1074/jbc.M114.553750 24713699PMC4022895

[B67] LarimoreJ.ZlaticS. A.ArnoldM.SingletonK. S.CrossR.RudolphH. (2017). Dysbindin deficiency modifies the expression of GABA neuron and ion permeation transcripts in the developing hippocampus. Front. Genet. 8, 28. 10.3389/fgene.2017.00028 28344592PMC5344932

[B68] LeeH. H.NemecekD.SchindlerC.SmithW. J.GhirlandoR.StevenA. C. (2012). Assembly and architecture of biogenesis of lysosome-related organelles complex-1 (BLOC-1). J. Biol. Chem. 287, 5882–5890. 10.1074/jbc.M111.325746 22203680PMC3285357

[B69] LeggioG. M.TorrisiS. A.MastrogiacomoR.MauroD.ChisariM.DevroyeC. (2019). The epistatic interaction between the dopamine D3 receptor and dysbindin-1 modulates higher-order cognitive functions in mice and humans. Mol. Psychiatry. 10.1038/s41380-019-0511-4 31492942

[B70] LemonnierE.LazartiguesA.Ben-AriY. (2016). Treating schizophrenia with the diuretic bumetanide: a case report. Clin. Neuropharmacol. 39, 115–117. 10.1097/WNF.0000000000000136 26966887

[B71] LewisD. A.HashimotoT.MorrisH. M. (2008). Cell and receptor type-specific alterations in markers of GABA neurotransmission in the prefrontal cortex of subjects with schizophrenia. Neurotox. Res. 14, 237–248. 10.1007/BF03033813 19073429PMC2884395

[B72] LiW.ZhangQ.OisoN.NovakE. K.GautamR.O’BrienE. P. (2003). Hermansky-Pudlak syndrome type 7 (HPS-7) results from mutant dysbindin, a member of the biogenesis of lysosome-related organelles complex 1 (BLOC-1). Nat. Genet. 35, 84–89. 10.1038/ng1229 12923531PMC2860733

[B73] LiW.RusiniakM. E.ChintalaS.GautamR.NovakE. K.SwankR. T. (2004). Murine Hermansky–Pudlak syndrome genes: regulators of lysosome-related organelles. Bioessays 26, 616–628. 10.1002/bies.20042 15170859

[B74] LucianoM.MiyajimaF.LindP. A.BatesT. C.HoranM.HarrisS. E. (2009). Variation in the dysbindin gene and normal cognitive function in three independent population samples. Genes Brain Behav. 8, 218–227. 10.1111/j.1601-183X.2008.00462.x 19077176

[B75] MalhotraD.SebatJ. (2012). CNVs: harbingers of a rare variant revolution in psychiatric genetics. Cell 148, 1223–1241. 10.1016/j.cell.2012.02.039 22424231PMC3351385

[B76] ManL.LvX.DuX. D.YinG.ZhuX.ZhangY. (2018). Cognitive impairments and low BDNF serum levels in first-episode drug-naive patients with schizophrenia. Psychiatry Res. 263, 1–6. 10.1016/j.psychres.2018.02.034 29482040

[B77] ManningB. D.CantleyL. C. (2007). AKT/PKB signaling: navigating downstream. Cell 129, 1261–1274. 10.1016/j.cell.2007.06.009 17604717PMC2756685

[B78] ManolioT. A.CollinsF. S.CoxN. J.GoldsteinD. B.HindorffL. A.HunterD. J. (2009). Finding the missing heritability of complex diseases. Nature 461, 747–753. 10.1038/nature08494 19812666PMC2831613

[B79] MarkW.ToulopoulouT. (2016). Cognitive intermediate phenotype and genetic risk for psychosis. Curr. Opin. Neurobiol. 36, 23–30. 10.1016/j.conb.2015.08.008 26363129

[B80] MarshallC. R.HowriganD. P.MericoD.ThiruvahindrapuramB.WuW.GreerD. S. (2017). Contribution of copy number variants to schizophrenia from a genome-wide study of 41,321 subjects. Nat. Genet. 49, 27–35. 10.1038/ng.3725 27869829PMC5737772

[B81] McCutcheonR. A.Abi-DarghamA.HowesO. D. (2019). Schizophrenia, dopamine and the striatum: from biology to symptoms. Trends Neurosci. 42, 205–220. 10.1002/wps.20693 30621912PMC6401206

[B82] MeierM. H.CaspiA.ReichenbergA.KeefeR. S.FisherH. L.HarringtonH. (2014). Neuropsychological decline in schizophrenia from the premorbid to the postonset period: evidence from a population-representative longitudinal study. Am. J. Psychiatry 171, 91–101. 10.1176/appi.ajp.2013.12111438 24030246PMC3947263

[B83] MullinA. P.SadanandappaM. K.MaW.DickmanD. K.VijayRaghavanK.RamaswamiM. (2015). Gene dosage in the dysbindin schizophrenia susceptibility network differentially affects synaptic function and plasticity. J. Neurosci. 35, 325–338. 10.1523/JNEUROSCI.3542-14.2015 25568125PMC4287151

[B84] NazarianR.StarcevicM.SpencerM. J.Dell’AngelicaE. C. (2006). Reinvestigation of the dysbindin subunit of BLOC-1 (biogenesis of lysosome-related organelles complex-1) as a dystrobrevin-binding protein. Biochem. J. 395, 587–598. 10.1042/BJ20051965 16448387PMC1462696

[B85] NumakawaT.YagasakiY.IshimotoT.OkadaT.SuzukiT.IwataN. (2004). Evidence of novel neuronal functions of dysbindin, a susceptibility gene for schizophrenia. Hum. Mol. Genet. 13, 2699–2708. 10.1093/hmg/ddh280 15345706

[B86] O’TuathaighC. M.WaddingtonJ. L. (2015). Closing the translational gap between mutant mouse models and the clinical reality of psychotic illness. Neurosci. Biobehav. Rev. 58, 19–35. 10.1016/j.neubiorev.2015.01.016 25616181

[B87] OwenM. J.SawaA.MortensenP. B. (2016). Schizophrenia. Lancet 388, 86–97. 10.1016/S0140-6736(15)01121-6 26777917PMC4940219

[B88] OyamaS.YamakawaH.SasagawaN.HosoiY.FutaiE.IshiuraS. (2009). Dysbindin-1, a schizophrenia-related protein, functionally interacts with the DNA-dependent protein kinase complex in an isoform-dependent manner. PloS One 4, e4199. 10.1371/journal.pone.0004199 19142223PMC2614472

[B89] PapaleoF.YangF.GarciaS.ChenJ.LuB.CrawleyJ. (2012). Dysbindin-1 modulates prefrontal cortical activity and schizophrenia-like behaviors *via* dopamine/D2 pathways. Mol. Psychiatry 7, 85–98. 10.1038/mp.2010.106 PMC338884820956979

[B90] PapaleoF.BurdickM. C.CallicottJ. H.WeinbergerD. R. (2014). Epistatic interaction between COMT and DTNBP1 modulates prefrontal function in mice and in humans. Mol. Psychiatry 19, 311–316. 10.1038/mp.2013.133 24145376PMC4845721

[B91] PetersK.WiltshireS.HendersA. K.DragovićM.BadcockJ. C.ChandlerD. (2008). Comprehensive analysis of tagging sequence variants in DTNBP1 shows no association with schizophrenia or with its composite neurocognitive endophenotypes. Am. J. Med. Genet. B Neuropsychiatr. Genet. 147B, 1159–1166. 10.1002/ajmg.b.30741 18314870

[B92] PetitE. I.MichalakZ.CoxR.O’TuathaighC. M.ClarkeN.TigheO. (2017). Dysregulation of specialized delay/interference-dependent working memory following loss of dysbindin-1A in schizophrenia-related phenotypes. Neuropsychopharmacology 42, 1349–1360. 10.1038/npp.2016.282 27986973PMC5437891

[B93] RahmanzadehR.EftekhariS.ShahbaziA.Khodaei ArdakaniM. R.RahmanzadeR.MehrabiS. (2017a). Effect of bumetanide, a selective NKCC1 inhibitor, on hallucinations of schizophrenic patients; a double-blind randomized clinical trial. Schizophr. Res. 184, 145–146. 10.1016/j.schres.2016.12.002 27956008

[B94] RahmanzadehR.ShahbaziA.ArdakaniM. K.MehrabiS.RahmanzadeR.JoghataeiM. T. (2017b). Lack of the effect of bumetanide, a selective NKCC1 inhibitor, in patients with schizophrenia: A double-blind randomized trial. Psychiatry Clin. Neurosci. 71, 72–73. 10.1111/pcn.12475 27800670

[B95] RammosA.GonzalezL. A. N.Schizophrenia Working Group of the Psychiatric Genomics ConsortiumWeinbergerD. R.MitchellK. J.NicodemusK. K. (2019). The role of polygenic risk score gene-set analysis in the context of the omnigenic model of schizophrenia. Neuropsychopharmacology. 10.1038/s41386-019-0410-z PMC678570731078131

[B96] RichardsA. L.PardiñasA. F.FrizzatiA.TanseyK. E.LynhamA. J.HolmansP. (2019). The relationship between polygenic risk scores and cognition in schizophrenia. Schizophr. Bull., pii: sbz061. 10.1093/schbul/sbz061 PMC744235231206164

[B97] SagguS.CannonT. D.JentschJ. D.LavinA. (2013). Potential molecular mechanisms for decreased synaptic glutamate release in dysbindin-1 mutant mice. Schizophr. Res. 146, 254–263. 10.1016/j.schres.2013.01.037 23473812PMC3628687

[B98] SavageJ. E.JansenP. R.StringerS.WatanabeK.BryoisJ.de LeeuwC. A. (2018). Genome-wide association meta-analysis in 269,867 individuals identifies new genetic and functional links to intelligence. Nat. Genet. 50, 912–919. 10.1038/s41588-018-0152-6 29942086PMC6411041

[B99] SchaeferJ.GiangrandeE.WeinbergerD. R.DickinsonD. (2013). The global cognitive impairment in schizophrenia: consistent over decades and around the world. Schizophr. Res. 150, 42–50. 10.1016/j.schres.2013.07.009 23911259PMC4196267

[B100] ScheggiaD.MastrogiacomoR.MereuM.SanninoS.StraubR. E.ArmandoM. (2018). Variations in Dysbindin-1 are associated with cognitive response to antipsychotic drug treatment. Nat. Commun. 9, 2265. 10.1038/s41467-018-04711-w 29891954PMC5995960

[B101] Schizophrenia Working Group of the Psychiatric Genomics Consortium (2014). Biological insights from 108 schizophrenia-associated genetic loci. Nature 511, 421–427. 10.1038/nature13595 25056061PMC4112379

[B102] ShaoL.ShuaiY.WangJ.FengS.LuB.LiZ. (2011). Schizophrenia susceptibility gene dysbindin regulates glutamatergic and dopaminergic functions *via* distinctive mechanisms in Drosophila. Proc. Natl. Acad. Sci. U.S.A. 108, 18831–18836. 10.1073/pnas.1114569108 22049342PMC3219129

[B103] ShintaniN.OnakaY.HashimotoR.TakamuraH.NagataT.Umeda-YanoS. (2014). Behavioral characterization of mice overexpressing human dysbindin-1. Mol. Brain 7, 74. 10.1186/s13041-014-0074-x 25298178PMC4201722

[B104] SillitoeR. V.BensonM. A.BlakeD. J.HawkesR. (2003). Abnormal dysbindin expression in cerebellar mossy fiber synapses in the mdx mouse model of Duchenne muscular dystrophy. J. Neurosci. 23, 6576–6585. 10.1523/JNEUROSCI.23-16-06576.2003 12878699PMC6740624

[B105] SinclairD.CesareJ.McMullenM.CarlsonG. C.HahnC. G.Borgmann-WinterK. E. (2016). Effects of sex and DTNBP1 (dysbindin) null gene mutation on the developmental GluN2B-GluN2A switch in the mouse cortex and hippocampus. J. Neurodev. Disord. 8, 14. 10.1186/s11689-016-9148-7 27134685PMC4852102

[B106] SpiegelS.ChiuA.JamesA. S.JentschJ. D.KarlsgodtK. H. (2015). Recognition deficits in mice carrying mutations of genes encoding BLOC-1 subunits pallidin or dysbindin. Genes Brain Behav. 14, 618–624. 10.1111/gbb.12240 26294018

[B107] StarcevicM.Dell’AngelicaE. C. (2004). Identification of snapin and three novel proteins (BLOS1, BLOS2, and BLOS3/reduced pigmentation) as subunits of biogenesis of lysosome-related organelles complex-1 (BLOC-1). J. Biol. Chem. 279, 28393–401.10.1074/jbc.M40251320015102850

[B108] StraubR. E.MacLeanC. J.O’NeillF. A.BurkeJ.MurphyB.DukeF. (1995). A potential vulnerability locus for schizophrenia on chromosome 6p24–22: evidence for genetic heterogeneity. Nat. Genet. 11, 287–293. 10.1038/ng1195-287 7581452

[B109] StrohmaierJ.FrankJ.WendlandJ. R.SchumacherJ.JamraR. A.TreutleinJ. (2010). A reappraisal of the association between Dysbindin (DTNBP1) and schizophrenia in a large combined case-control and family-based sample of German ancestry. Schizophr. Res. 118, 98–105. 10.1016/j.schres.2009.12.025 20083391PMC2856768

[B110] SullivanC. R.FunkA. J.ShanD.HaroutunianV.McCullumsmithR. E. (2015). Decreased chloride channel expression in the dorsolateral prefrontal cortex in schizophrenia. PloS One 10, e0123158. 10.1371/journal.pone.0123158 25826365PMC4380350

[B111] StraubR. E.MayhewM. B.VakkalankaR. K.KolachanaB.GoldbergT. E.EganM. F. (2005). MUTED, a protein that binds to dysbindin (DTNBP1), is associated with schizophrenia. Am. J. Med. Genet. B Neuropsychiatr. Genet. 138B, 136.

[B112] SwankR. T.SweetH. O.DavissonM. T.ReddingtonM.NovakE. K. (1991). Sandy: a new mouse model for platelet storage pool deficiency. Genet. Res. 58, 51–62. 10.1017/s0016672300029608 1936982

[B113] TakaoK.ToyamaK.NakanishiK.HattoriS.TakamuraH.TakedaM. (2008). Impaired long-term memory retention and working memory in sdy mutant mice with a deletion in Dtnbp1, a susceptibility gene for schizophrenia. Mol. Brain 1, 11–23. 10.1186/1756-6606-1-11 18945333PMC2584096

[B114] TalbotK.EidemW. L.TinsleyC. L.BensonM. A.ThompsonE. W.SmithR. J. (2004). Dysbindin-1 is reduced in intrinsic, glutamatergic terminals of the hippocampal formation in schizophrenia. J. Clin. Invest. 113, 1353–1363. 10.1172/JCI20425 15124027PMC398430

[B115] TalbotK.ChoD.-S.OngW.-Y.BensonM. A.HanL.-Y.KaziH. A. (2006). Dysbindin-1 is a synaptic and microtubular protein that binds brain snapin. Hum. Mol. Genet. 15, 3041–3054. 10.1093/hmg/ddl246 16980328

[B116] TalbotK.LounevaN.CohenJ. W.KaziH.BlakeD. J.ArnoldS. E. (2011). Synaptic dysbindin-1 reductions in schizophrenia occur in an isoform-specific manner indicating their subsynaptic location. PloS One 6, e16886. 10.1371/journal.pone.0016886 21390302PMC3046962

[B117] TalbotK. (2009). The sandy (sdy) mouse: a dysbindin-1 mutant relevant to schizophrenia research. Prog.Brain Res. 179, 87–94. 10.1016/S0079-6123(09)17910-4 20302821

[B118] TamV.PatelN.TurcotteM.BosséY.ParéG.MeyreD. (2019). Benefits and limitations of genome-wide association studies. Nat. Rev. Genet. 20, 467–484. 10.1038/s41576-019-0127-1 31068683

[B119] TammingaC. A.StanA. D.WagnerA. D. (2010). The hippocampal formation in schizophrenia. Am. J. Psychiatry 167, 1178–1193. 10.1176/appi.ajp.2010.09081187 20810471

[B120] Taneichi-KurodaS.TayaS.HikitaT.FujinoY.KaibuchiK. (2009). Direct interaction of Dysbindin with the AP-3 complex *via* its mu subunit. Neurochem. Int. 54, 431–438. 10.1016/j.neuint.2009.01.014 19428785

[B121] TangJ.LeGrosR. P.LounevaN.YehL.CohenJ. W.HahnC.-G. (2009). Dysbindin-1 in dorsolateral prefrontal cortex of schizophrenia cases is reduced in an isoform-specific manner unrelated to dysbindin-1 mRNA expression. Hum. Mol. Genet. 18, 3851–3863. 10.1093/hmg/ddp329 19617633PMC2748893

[B122] TanseyK. E.ReesE.LindenD. E.RipkeS.ChambertK. D.MoranJ. L. (2016). Common alleles contribute to schizophrenia in CNV carriers. Mol. Psychiatry 21, 1153. 10.1038/mp.2015.170 PMC760934426643540

[B123] ToulopoulouT.ZhangX.ChernyS.DickinsonD.BermanK. F.StraubR. E. (2019). Polygenic risk score increases schizophrenia liability through cognition-relevant pathways. Brain 142, 471–485. 10.1093/brain/awy279 30535067PMC6359897

[B124] Varela-GomezN.MataI.Perez-IglesiasR.Rodriguez-SanchezJ. M.AyesaR.Fatjo-VilasM. (2015). Dysbindin gene variability is associated with cognitive abnormalities in first-episode non-affective psychosis. Cogn. Neuropsychiatry 20, 144–56. 10.1080/13546805.2014.991780 25530342

[B125] VijayraghavanS.WangM.BirnbaumS. G.WilliamsG. V.ArnstenA. F. (2007). Inverted-U dopamine D1 receptor actions on prefrontal neurons engaged in working memory. Nat. Neurosci. 10, 376–384. 10.1038/nn1846 17277774

[B126] WaddingtonJ. L.HennessyR. J.O’TuathaighC. M. P.OwoeyeO.RussellV. (2012). Schizophrenia and the lifetime trajectory of psychotic illness: developmental neuroscience and pathobiology, redux, in The origins of schizophrenia. Eds. BrownA. S.PattersonP. H. (New York: Columbia University Press), pp. 3–21.

[B127] WangH.XuJ.LazaroviciP.ZhengW. (2017). Dysbindin-1 involvement in the etiology of schizophrenia. Int. J. Mol. Sci. 18, pii: E2044. 10.3390/ijms18102044 PMC566672628937620

[B128] WangP.CaoT.ChenJ.JiangY.WangC.WaddingtonJ. L. (2019). D2 receptor-mediated miRNA-143 expression is associated with the effects of antipsychotic drugs on phencyclidine-induced schizophrenia-related locomotor hyperactivity and with neuregulin-1 expression in mice. Neuropharmacology. 157, 107675. 10.1016/j.neuropharm.2019.107675 31233824

[B129] WeickertC. S.StraubR. E.McClintockB. W.MatsumotoM.HashimotoR.HydeT. M. (2004). Human dysbindin (DTNBP1) gene expression in normal brain and in schizophrenic prefrontal cortex and midbrain. Arch. Gen. Psychiatry 61, 544–545. 10.1001/archpsyc.61.6.544 15184234

[B130] WeickertC. S.RothmondD. A.HydeT. M.KleinmanJ. E.StraubR. E. (2008). Reduced DTNBP1 (dysbindin-1) mRNA in the hippocampal formation of schizophrenia patients. Schizophr. Res. 98, 105–110. 10.1016/j.schres.2007.05.041 17961984PMC2246024

[B131] WeinbergerD. R. (2017). Future of days past: neurodevelopment and schizophrenia. Schizophr. Bull. 43, 1164–1168. 10.1093/schbul/sbx118 29040792PMC5737209

[B132] WeinbergerD. R. (2019). Thinking about schizophrenia in an era of genomic medicine. Am. J. Psychiatry 176, 12–20. 10.1176/appi.ajp.2018.18111275 30848926

[B133] XavierR. M.DunganJ. R.KeefeR. S. E.VorderstrasseA. (2018). Polygenic signal for symptom dimensions and cognitive performance in patients with chronic schizophrenia. Schizophr. Res. Cogn. 12, 11–19. 10.1016/j.scog.2018.01.001 29552508PMC5852279

[B134] XuY.SunY.YeH.ZhuL.LiuJ.WuX. (2015). Increased dysbindin-1B isoform expression in schizophrenia and its propensity in aggresome formation. Cell. Discovery 1, 15032. 10.1038/celldisc.2015.32 27462430PMC4860834

[B135] YangW.XuQ. (2017). Hippocampal apoptosis and cognitive function in Dysbindin-1B mice. Zhongguo Yi Xue Ke Xue Yuan Xue Bao. 39, 307–311. 10.3881/j.issn.1000-503X.2017.03.002 28695798

[B136] YangW.ZhuC.ShenY.XuQ. (2016). The pathogenic mechanism of dysbindin-1B toxic aggregation: BLOC-1 and intercellular vesicle trafficking. Neuroscience 333, 78–91. 10.1016/j.neuroscience.2016.07.008 27421225

[B137] YangY.LiuY.WangG.HeiG.WangX.LiR. (2019). Brain-derived neurotrophic factor is associated with cognitive impairments in first-episode and chronic schizophrenia. Psychiatry Res. 273, 528–536. 10.1016/j.psychres.2019.01.051 30710808

[B138] ZhangJ. P.BurdickK. E.LenczT.MalhotraA. K. (2010). Meta-analysis of genetic variation in DTNBP1 and general cognitive ability. Biol. Psychiatry 68, 1126–1133. 10.1016/j.biopsych.2010.09.016 21130223PMC3026311

[B139] ZhengW.WangH.ZengZ.LinJ.LittleP. J.SrivastavaL. K. (2012). The possible role of the Akt signaling pathway in schizophrenia. Brain Res. 1470, 145–148. 10.1016/j.brainres.2012.06.032 22771711

